The article "Correlation between Pain Scores and Disc Height Changes after Discectomy in Patients with Lumbar Disc Herniation: A Systematic Review and Meta-Analysis" was retracted in 2023. Reasons: unreliable results or conclusions; concerns about the data; concerns about the peer review; concerns about the citations.

# Correlation between Pain Scores and Disc Height Changes after Discectomy in Patients with Lumbar Disc Herniation: A Systematic Review and Meta-Analysis

**DOI:** 10.1155/2022/2580004

**Published:** 2022-08-05

**Authors:** Yuchen Zheng, Tao Lan, Xiaosheng Chen, Zhihao Hus, Rui Zhang

**Affiliations:** Department of Spine Surgery, Shenzhen Second People's Hospital, The First Affiliated Hospital of Shenzhen University, Shenzhen 518035, China

## Abstract

**Background:**

Surgery can reduce and improve lumbar disc herniation, but some patients still have pain after surgery, and the relationship between lumbar disc height and pain after surgery is still unclear.

**Objective:**

The main objective is to investigate the relationship between lumbar disc height and postoperative pain.

**Methods:**

We searched Pubmed, Web of Science, the Cochrane library, and Embase online for cohort studies or RCT studies on discectomy and assessed the quality of the included articles using the Newcastle-Ottawa Scale (NOS scale), with disc height (DH) and postoperative back pain as the main clinical outcome indicators, and the correlation coefficient between DH and back pain as the statistic to assess the pooled effect size.

**Results:**

10 kinds of literature were included in this study for quantitative analysis. A total of 589 patients participated in the study. The follow-up time was between 1 and 2.3 years. Meta-analysis showed that after surgery, the relief of back pain was statistically significant (*MD* = −2.57, 95% CI (−3.10,−2.04), *Z* = −9.570, *P* < 0.0001), the reduction of disc height was statistically significant (*MD* = −0.82, 95% CI (−1.11, −0.52), *Z* = −5.477, *P* < 0.0001), the combined value of correlation coefficient Fisher's *Z* value was 0.33, 95% CI (0.25,0.42), with statistical significance (*P* < 0.00001), suggesting that the degree of back pain after surgery showed a moderate positive correlation with disc height in the short term. *Discussion*. After discectomy, the degree of pain is relieved, the disc height is reduced, and low back pain in the short term and disc height showed a moderate positive correlation, but the long-term correlation remains to be studied in depth.

## 1. Introduction

Lumbar disc herniation (LDH) is a common spinal disorder with low back and leg pain in the elderly. The cause is degeneration of the lumbar disc, which ruptures the annular fibers, exposes the nucleus pulposus, compresses nerve bundles, and causes persistent pain [1]. Lumbar disc herniation is clinically presented as a syndrome of lumbar and leg pain, and degenerative changes in intervertebral discs, trauma, pregnancy, and even heredity can cause its onset. For patients with mild symptoms, nonsurgical treatment (physical therapy, drug therapy, diet modification, lifestyle changes) is preferred, but for patients with severe symptoms, recurrent attacks, and ineffective treatment with nonsurgical methods, minimally invasive spinal techniques can be considered, and especially, endoscopic spinal surgery is recommended [2]. Despite the excellent clinical outcome of surgery, it has been reported that 30% of patients still have low back pain (LBP) [3]. Factors such as unreasonable choice of surgical patients, unclear diagnosis, and outdated surgical instruments or techniques may be related to persistent postoperative low back pain, but the exact cause is unclear [4]. As the partially herniated nucleus pulposus tissue is removed in lumbar discectomy, the loss of intervertebral disc height (DH) or even lumbar instability may occur after the operation, or it may accelerate the degeneration process of surgery and cause the recurrence of low back pain or LDH [5]. Some studies [6] have shown that decreased DH after lumbar discectomy may be one of the causes of long-term low back and leg pain. However, some studies [7] suggested that the decrease in intervertebral disc height in a short period of time contributed to the alleviation of pain, and in order to understand the correlation between DH and low back pain after lumbar discectomy, we performed this meta-analysis.

The article "Correlation between Pain Scores and Disc Height Changes after Discectomy in Patients with Lumbar Disc Herniation: A Systematic Review and Meta-Analysis" was retracted in 2023. Reasons: unreliable results or conclusions; concerns about the data; concerns about the peer review; concerns about the citations.

## 2. Materials and Methods

### 2.1. Database and Search Strategy

We searched Pubmed, Web of Science, the Cochrane library, and Embase online for the literature related to discectomy. We only included the literature published in the past 10 years from January 2011 to November 2021. The electronic search was performed with the keyword combination [*discectomy*] AND/OR [*lumbar disc herniation*] AND/OR [*lumbar spine*] AND/OR [*percutaneous discectomy*]. We set the screening criteria and screened the retrieved literature.

### 2.2. Literature Inclusion Criteria

(1) *Study Type*: all kinds of literature were observational studies or RCT literature, regardless of whether the research process uses blinding or not. For RCT literature, we only included one group related to discectomy in the random grouping into statistical analysis, and we did not limit the literature to prospective or retrospective cohort study; (2) *Study Subjects*: all patients were treated with disc herniation; (3) *Intervention Type*: all patients received discectomy for surgical intervention, and we did not limit the types of surgery to percutaneous endoscopic lumbar discectomy (PLED), microendoscopic discectomy (MED), or conventional lumbar discectomy (CLD) and did not limit the implantation of an annular closure device during surgery. (4) *Outcome Indicators*: we only included the literature reporting the intervertebral disc height (DH) and postoperative back pain. In order to eliminate the heterogeneity of indicator assessment, the way to assess the pain must be reported only by VAS (Visual Analogue Scale). The short term is defined as no more than 1 month after the operation, and the long term is defined as after 1 month after the operation. The VAS score data included in the literature contain or can be extrapolated mean and standard deviation.

The article "Correlation between Pain Scores and Disc Height Changes after Discectomy in Patients with Lumbar Disc Herniation: A Systematic Review and Meta-Analysis" was retracted in 2023. Reasons: unreliable results or conclusions; concerns about the data; concerns about the peer review; concerns about the citations.

### 2.3. Literature Exclusion Criteria

(1) We excluded all case-control studies, individual case studies, reviews, and meeting minutes. (2) We excluded patients whose study subjects are cervical discectomy. (3) We excluded studies that lack outcome indicators, or have no data. Lumbar disc herniation was excluded as a multisegment herniation, with a history of lumbar spine surgery, and diseases affect the evaluation of efficacy such as vertebral instability, spinal deformity, spinal stenosis, and severe osteoporosis. The types of excluded literature are reviews, animal experiments, conference papers, and repeated publications. (4) VAS scores designated as parts of the body (e.g., waist, legs) should be excluded. Studies with incomplete literature data and no access to authors in the associated literature should be excluded.

### 2.4. Literature Screening

The screened literature was imported into the software Note express for unified management after retrieval and manual removal. The deduplication function of the software was used to exclude repeated literature. 2 researchers read the title and abstract for further screening. The screening results were cross-checked and discussed to determine the selected literature. If the original text could not be obtained from the Internet, the author of the original text was contacted by telephone or e-mail; if the original text could not be obtained, the literature was excluded.

### 2.5. Literature Quality Evaluation and Risk of Bias Assessment

The Newcastle-Ottawa Scale (NOS scale) [8] was used to analyze the quality of the included literature. The scale was used to evaluate the object selection, comparability, and outcome indicators of the literature. The maximum score was 9 points. The score of more than 5 points was considered good quality. The higher the score, the better the literature quality and the less bias.

### 2.6. Data Extraction and Analysis

2 researchers independently extracted literature data: study type, location, patient age, height, weight, surgical method, surgical site, number of cohorts, follow-up time, and outcome indicators. After data extraction by 2 researchers, the results of each other were cross-checked, and the differences generated were discussed and finally determined.

The article "Correlation between Pain Scores and Disc Height Changes after Discectomy in Patients with Lumbar Disc Herniation: A Systematic Review and Meta-Analysis" was retracted in 2023. Reasons: unreliable results or conclusions; concerns about the data; concerns about the peer review; concerns about the citations.

### 2.7. Outcome Indicators

The main outcome indicators were the height of intervertebral disc height and the degree of back pain after operation (BP-VAS). There was no fixed standard for the calculation method of intervertebral disc height. We counted the DH calculation method included in the study and tried to analyze whether it would bring heterogeneity. The correlation coefficient between DH and BP-VAS in the literature was expressed by Pearson's correlation coefficient *γ*, and if not given directly in the literature, we will contact the original authors and calculate the correlation coefficient after obtaining the raw data. The significance of the values of the correlation coefficient *γ* is a very strong correlation, 0.8–1.0; strong correlation, 0.6–0.8; moderate intensity correlation, 0.4–0.6; weak correlation, 0.2–0.4; no correlation, 0–0.2.

### 2.8. Data Conversion

Before performing a meta-analysis of correlation coefficients, we need to convert the data (correlation coefficients *γ*), calculate Fisher's *Z* value and its *SE* value, and then import into meta-analysis software for inverse variance analysis [9]. The conversion formula is as follows:

(1) $$\begin{array}{c} \text{fisher}\prime s\;Z=0.5\times \;\ln\frac{1+\gamma }{1-\gamma },\\ Vz=\frac{1}{n-3},\\ S\varepsilon =\sqrt{Vz}. \end{array}$$

### 2.9. Statistical Methods

(a) We used both STATA 16.0 (released by STATA Corp LLC) and Revman 5.3 (released by The Nordic Cochrane Centre, The Cochrane Collaboration, 2014) for analysis; (b) continuous variables were reported using mean difference (*SMD*) and 95% CI statistics, using STATA 16.0 software to analyze; (c) correlation coefficient analysis inputs Fisher's *Z* statistics and *Se* value after correlation coefficient *γ* conversion into Revman 5.3 software. The inverse variance was used for analysis, and the forest plot descriptive statistics were used for comparison. (d) The *I*^*2*^ analysis and *Q* test were used for literature heterogeneity. The *I*^*2*^ > 50% or *P* < 0.1 indicated heterogeneity of the results. The random-effect model was used to obtain the *SMD* value, and otherwise, the fixed-effect model was used to obtain the *SMD* value; (e) if the heterogeneity analysis suggested heterogeneity between the kinds of literature, the subgroup analysis investigated the heterogeneity source. When the heterogeneity source could not be determined, the general description was adopted; (f) the funnel plot was used to represent the publication bias.

## 3. Results

### 3.1. Literature Screening Process and Results

Figure 1 shows the flow chart of literature selection, and finally, 10 kinds of literature were included in the quantitative analysis, with a total of 589 patients participating in the study.

The article "Correlation between Pain Scores and Disc Height Changes after Discectomy in Patients with Lumbar Disc Herniation: A Systematic Review and Meta-Analysis" was retracted in 2023. Reasons: unreliable results or conclusions; concerns about the data; concerns about the peer review; concerns about the citations.

### 3.2. Basic Characteristics of Literature

Ten kinds of literature were included in this study, including 4 retrospective cohort studies, 5 prospective cohort studies, and 1 RCT study. The minimum follow-up time was 1 year, and the maximum follow-up time was 2.3 years. The details are shown in Table 1.

### 3.3. Literature Quality and Bias Evaluation

In this study, all the included cases in the literature [10–19] were representative, with a less potential risk of bias. Some literature [14–16] did not describe the baseline data, and some literature did not describe the drop-out cases in detail [11,12,14–17,19]. However, the overall quality score of all literature was 7–9 points, with good quality, as shown in Table 2.

### 3.4. Meta-Analysis Results

#### 3.4.1. Changes in the Degree of Pain (back) before and after Lumbar Discectomy

All literature [10–19] reported the back pain severity (BP-VAS). Meta-analysis was performed using random-effect model. After the surgery, the back pain was significantly relieved, with statistical significance (*MD* = −2.57, 95% CI (−3.10,−2.04), *Z* = −9.570, *P* < 0.0001).

Further subgroup analysis of the literature according to the surgical method or DH calculation method showed that there was still heterogeneity among the internal literature, but the degree of back pain relief was statistically significant among the literature (*P* < 0.0001), as shown in Figures 2 and 3.

#### 3.4.2. Changes in Disc Height before and after Lumbar Discectomy (mm)

All literature [10–19] reported the change in disc height before and after the operation. The random-effects model analysis was used to obtain that the disc height decreased after the operation. The decrease was statistically significant (*MD* = −0.82, 95% CI (−1.11, −0.52), *Z* = −5.477, *P* < 0.0001).

Further subgroup analysis of the literature according to the surgical method or DH calculation method showed that there was still heterogeneity among the internal literature, and the decrease in disc height before and after the surgery was statistically significant (*P* < 0.0001), as shown in Figures 4 and 5.

#### 3.4.3. Meta-Correlation Coefficient Analysis between the Degree of (back) Pain and Disc Height

There was no statistical heterogeneity in the reported correlation coefficient between the 10 included literature (*I*^*2*^ = 0%, *P*=0.46). Fixed-effect model was used, and meta-analysis showed that the combined value of the correlation coefficient Fisher's *Z* was 0.33, 95% CI (0.25, 0.42), with statistical significance (*P* < 0.0001), suggesting that there was a moderate positive correlation between the degree of back pain after surgery and disc height as shown in Figure 6.

The article "Correlation between Pain Scores and Disc Height Changes after Discectomy in Patients with Lumbar Disc Herniation: A Systematic Review and Meta-Analysis" was retracted in 2023. Reasons: unreliable results or conclusions; concerns about the data; concerns about the peer review; concerns about the citations.

#### 3.4.4. Source of Heterogeneity and Sensitivity Analysis

In the analysis of the change indicator of disc height before and after the operation, there was statistical heterogeneity between the kinds of literature (*I*^*2*^ = 82.4%, *P*=0.01). After the kinds of literature were divided into subgroups according to the operation method and DH calculation method, the internal heterogeneity was not eliminated. We speculated that the existence of heterogeneity may be related to multiple factors such as patient age level, disease type, operation method, and follow-up time.

In the correlation coefficient analysis, the random-effects model was used, and the results were similar to those of the fixed-effects model, showing that the results had good stability (good sensitivity).

#### 3.4.5. Publication Bias Analysis

In the analysis of the correlation coefficient, the funnel plot shows that the two sides of the funnel are basically evenly distributed, suggesting that the publication bias is small, as shown in Figure 7.

## 4. Discussion

In this meta-analysis, we retrieved and identified 10 related articles with a total of 589 patients who underwent 2 types of surgery: PLED or CLD. All kinds of literature reported lower back pain (VAS) and disc height value. All patients had statistically significant pain relief and DH value reduction by comparing the data before and after the operation. We tried to analyze the kinds of literature. 221 patients underwent PLED surgery in 4 kinds of literature, 368 patients underwent CLD surgery in 6 literature. 5 kinds of literature used Method 1 DH calculation method, 2 kinds of literature used Method 2, 2 kinds of literature used Method 3, and 1 literature used Method 4. All blood pressure-VAS and DH statistical results show that pain relief can be achieved regardless of which discectomy is used, and disc height is reduced in any surgical method. The study by Orpen et al. [20] concluded that the nucleus pulposus tissue is a gelatinous semiliquid substance with some fluidity. After a discectomy to remove a part of the nucleus pulposus tissue, the original integrity of the intervertebral disc has been damaged. The intervertebral disc capacity will gradually show degeneration and absorption phenomenon, so that the overall structure formed by the intervertebral disc and the upper and lower vertebral bodies are damaged. The height of the lesion space naturally decreases, which makes the intervertebral disc height decrease accordingly.

The article "Correlation between Pain Scores and Disc Height Changes after Discectomy in Patients with Lumbar Disc Herniation: A Systematic Review and Meta-Analysis" was retracted in 2023. Reasons: unreliable results or conclusions; concerns about the data; concerns about the peer review; concerns about the citations.

In this meta-analysis, we performed a summary of Fisher's *Z* transformation on the correlation coefficient *γ* between lower back pain (VAS) and disc height reported in each literature, and Revman's pooling was performed using the inverse variance method and presented in a forest plot, resulting in a fisher's *Z* pooling was 0.33, 95% CI (0.25,0.42), which was statistically significant (*P* < 0.00001), and the forest plot showed that there was a moderately strong correlation between lower back pain and disc height values. Studies [21] have shown that after discectomy, the destruction of vertebral annular integrity leads to significant changes in disc pressure and changes in disc height, which may be related to the amount of resection and the degree of disc bulging. A decrease in DH may lead to a decrease in the relative movement between the vertebrae, which can quickly reduce exercise-related pain [22]. However, with the decrease in the height of the intervertebral disc, the anterior and posterior longitudinal ligaments of the intervertebral disc become relaxed, and the range of motion of the lumbar spine increases, which may lead to adhesions and hyperplasia of the small joints, thus affecting the stability of the lumbar spine [23]. In the long term, decreased intradiscal pressure and increased facet loading after the loss of DH after discectomy have the potential to have adverse effects on the stability of the spine, increasing postoperative pain scores[24]. However, there are also some shortcomings in this study, as the maximum follow-up time of the studies we included was 2.3 years and no long-term follow-up was studied, so there are still some limitations to the correlation between lower back pain (VAS) and intervertebral disc height values.

10 RCTs were included in this study. The total score of the NOS methodology assessment was more than 7 points, with good quality. During subgroup analysis, heterogeneity was still shown in the 2 groups, which may be related to multiple factors such as patient age level, disease type, surgical method, and follow-up time. However, for the analysis of the correlation coefficient between the lower back pain (VAS) and disc height value, there was no heterogeneity among the literature, and the results were stable. The funnel plot showed that the distribution on both sides was symmetrical, suggesting that the publication bias was small. However, this study did not include long-term follow-up studies, and the study on this topic still needs to be further explored in terms of sample size.

## 5. Conclusion

This meta-analysis included 10 literature with a total of 589 patients. The results showed that the pain was relieved after discectomy, and the intervertebral disc height was reduced. There was a moderate positive correlation between low back pain and intervertebral disc height in a short period of time. However, the long-term correlation remains to be further studied.

The article "Correlation between Pain Scores and Disc Height Changes after Discectomy in Patients with Lumbar Disc Herniation: A Systematic Review and Meta-Analysis" was retracted in 2023. Reasons: unreliable results or conclusions; concerns about the data; concerns about the peer review; concerns about the citations.

## Figures and Tables

**Figure 1:** Literature selection flow chart.

**Figure 2:** Changes in the degree of back pain before and after discectomy (grouped by surgical method).

**Figure 3:** Changes in the degree of back pain before and after discectomy (grouped according to DH calculation method).

**Figure 4:** Changes of disc height before and after discectomy (grouped by surgical method).

**Figure 5:** Changes in disc height before and after discectomy (grouped by DH calculation method).

**Figure 6:** Correlation analysis between the degree of back pain after discectomy and disc height.

**Figure 7:** Funnel plot analysis.

**Table 1:** Basic characteristics, intervention measures, intervention time and outcome indicators of the included literature.

Author and date of publication	Study design	Mean age (year)	Patients number	Surgery type	Surgery level	Follow-up time	DH method	Correlation coefficient *γ*	Outcomes
Ren C [10]	Prospective cohort study	45.6 ± 12.2	54	PELD	L3-L4; L4-L5; L5-S1	1 years	Method 1	0.338	1/2/3/4/5

Choi KC [11]	Retrospective cohort study	38.3 ± 10.3	100	PELD	L5-S1	2 years	Method 2	0.464	1/2/3/5

Lee JH [12]	Prospective cohort study	48.6 ± 6.3	42	PELD	L3-L4; L4-L5; L5-S1	1 years	Method 1	0.255	1/2/3/4/5

Cho PG [13]	RCT	42.6 ± 11.5	30	CLD	L3-L4; L4-L5; L5-S1	1 years	Method 1	0.521	1/2/3/4/5

Wu Q [14] 2021	Prospective cohort study	46.2 ± 12	100	CLD	L3-L4; L4-L5; L5-S1	1.1 years	Method 1	0.335	1/2/3/4/5

Li Z [15]	Retrospective cohort study	38	72	CLD	L3-L4; L4-L5; L5-S1	2.3 years	Method 1	0.128	1/2/3/4/6

Lequin MB [16]	Prospective cohort study	42.3 ± 11.4	45	CLD	L3-L4; L4-L5; L5-S1	1 years	Method 3	0.299	1/2/3/5

Ledic D [17]	Retrospective cohort study	38.3 ± 9.5	75	CLD	L3-L4; L4-L5; L5-S1	2 years	Method 3	0.235	1/2/3/5

Parker SL [18]	Prospective cohort study	38 ± 9	46	CLD	N/A	2 years	Method 2	0.233	1/2/3/6

Luo K [19]	Retrospective cohort study	45.6 ± 10.9	25	PELD	L3-L4; L4-L5; L5-S1	1 years	Method 4	0.410	1/2/3/6

Outcomes: 1. back pain (VAS); 2. leg pain (VAS); 3. ODI score; 4. SF36 score; 5. disc height; 6. JOA score. DH method: Method 1 - the (anterior + posterior disc height)/2; Method 2 - the vertical distance between the posterior lower plate of the L5 vertebral body (VB) and the posterior upper plate of the sacrum; Method 3 - the distance between the anterior-inferior corner of the superior vertebra and the corresponding corner of the inferior vertebra. Method 4 - the (anterior disc height + central disc height + posterior disc height)/3. Abbreviations. PLED-percutaneous endoscopic lumbar discectomy. CLD-conventional lumbar discectomy. ODI - the Oswestry disability Index. JOA - Japanese orthopaedic association (JOA) score. N/A- not available.

The article "Correlation between Pain Scores and Disc Height Changes after Discectomy in Patients with Lumbar Disc Herniation: A Systematic Review and Meta-Analysis" was retracted in 2023. Reasons: unreliable results or conclusions; concerns about the data; concerns about the peer review; concerns about the citations.

**Table 2:** Quality assessment based on Newcastle-Ottawa scale (NOS).

Study	Case selection (/4)	Comparability (/2)	Outcome indicators (/3)	Total score (/9)
Ren C [10]	4	2	3	9
Choi KC [11]	4	2	2	8
Lee JH [12]	4	2	2	8
Cho PG [13]	4	2	3	9
Wu *Q* [14]	4	1	2	7
Li Z [15]	4	1	2	7
Lequin MB [16]	4	1	2	7
Ledic D [17]	4	2	2	8
Parker SL [18]	4	2	3	9
Luo K [19]	4	2	2	8

## Data Availability

No data were used to support this study.
